# Meta-Analysis of the Effect of Dietary Care on Nausea and Vomiting in Oncology Chemotherapy Patients

**DOI:** 10.1155/2022/3163230

**Published:** 2022-07-31

**Authors:** Jing He, Ying Xiong, Dong Mo, Min Tang

**Affiliations:** Department of Oncology, Chongqing General Hospital, Chongqing 401147, China

## Abstract

**Objective:**

To evaluate the effect of dietary care on chemotherapy-induced nausea and vomiting in oncology patients.

**Methods:**

A retrospective analysis of digestive symptoms was conducted in cancer patients admitted to our hospital, who received chemotherapy, and corresponding effective dietary care countermeasures were adopted.

**Results:**

After the nursing intervention, the incidence of digestive symptoms was significantly reduced, the quality of life was significantly improved (59.92 ± 6.57) vs. (37.95 ± 7.50), and the nursing satisfaction was significantly higher (91.67% vs. 69.44%), with statistically significant differences (*P* < 0.05). Meta-analysis showed that short-term (0 to 3 months) dietary care could alleviate nausea and vomiting symptoms in chemotherapy patients (*P* < 0.001) and improve the survival quality of oncology patients (*P* < 0.01). The effect of long-term (3–6 months) dietary care on the control of nausea and vomiting symptoms in chemotherapy patients was certain (*P* < 0.05), but the effect on the improvement of their quality of life (*P* > 0.05) was unclear.

**Conclusion:**

Dietary care can alleviate the symptoms of nausea and vomiting in tumor chemotherapy patients and improve the quality of life of short-term chemotherapy tumor patients, so it can be recommended to strengthen the dietary management for tumor patients receiving chemotherapy. Patients receiving chemotherapy should be given corresponding dietary nutritional care according to their clinical symptoms in order to alleviate their adverse reactions, enhance their own immunity, and improve the prognosis of cancer patients.

## 1. Introduction

A good diet can provide cancer patients with reasonable and adequate nutrition and strengthen their own immunity, thus enhancing their ability to fight against the adverse effects of cancer treatment [1]. In particular, gynecologic malignant tumors are common gynecologic diseases in women, which have a serious impact on patients' physical and mental health and quality of life, and even threaten their life safety. At present, chemotherapy is mainly used in clinical practice for corresponding treatment, and chemotherapy operation may cause malnutrition in patients, so how to take effective measures to intervene and improve patients' nutritional status tests the practical ability of nursing staff [2–4].

Malignant tumor has become an important disease threatening human health. A total of 12.66 million new malignant tumor patients and 7.6 million deaths were reported worldwide in 2008 [5], and by 2030, the number of deaths will rise to 11.4 million and leap to the second place in global disease mortality [6]. Chemotherapy, as an important treatment for malignant tumors, kills cancer cells and also kills normal cells that are actively proliferating in the body. Among many chemotherapy-sensitive tissues in the human body, the digestive tract is one of the first to be affected [7]. Tumor patients suffer from different degrees of GI damage during chemotherapy, and these adverse reactions seriously reduce patients' chemotherapy tolerance and survival quality [8], and among many GI toxic reactions, nausea and vomiting are the most common. Severe vomiting can lead to loss of appetite, disturbance of water, electrolyte, acid-base balance, decreased immunity and other reactions, and the patient's nervousness and anxiety [9].

At present, chemotherapy has a large proportion in the treatment of gynecologic malignancies, which can significantly improve the survival of patients, but there are many side effects of chemotherapy drugs, which can lead to serious adverse effects on the metabolic function of the body and cause malnutrition, which has a significant impact on the physical and mental health of patients [10]. Providing chemotherapy dietary guidance to patients is the main method to improve their nutritional status. Some literature [11] reported that malnutrition is an independent risk factor for the prognosis of patients with malignant tumors, and the tolerance of chemotherapy treatment is significantly reduced after the occurrence of malnutrition. Dietary intervention can provide scientific guidance to patients' chemotherapy diet, improve malnutrition, and avoid the occurrence of impaired absorption and metabolism of chemotherapy drugs [12–15].

After the dietary intervention, the nutritional indexes of the cases in the observation group selected in this study improved significantly, and the patient care satisfaction was higher than that of the patients in the conventional care group. In other words, giving systematic dietary interventions can improve the nutritional status of patients with gynecological malignancies and promote the smooth development of chemotherapy treatment [16–18].

Despite the routine use of antiemetics during clinical treatment, the control of nausea and vomiting in chemotherapy patients is not optimistic. From basic experimental mechanism exploration to clinical practice verification, studies on dietary care to alleviate chemotherapy-induced nausea and vomiting have been increasing in recent years, but no analytical evaluation of the relevant literature has been seen. The purpose of this systematic evaluation is to evaluate the efficacy of dietary interventions for the relief of nausea and vomiting after chemotherapy and to provide evidence to support the development of clinical care protocols by summarizing the literature of relevant randomized controlled trials at home and abroad.

## 2. Materials and Methods

### 2.1. General Information

Eighty-six patients with gynecological malignancies were selected as observation subjects, and all selected patients met the criteria for disease diagnosis and treatment [1], and the patients had no consciousness disorders and were able to cooperate with the treatment work. According to the grouping of nursing methods, the observation group (*n* = 43) was aged 38 to 67 years, with an average age of (43.63 ± 3.58) years. The control group was 37–68 years old, with a mean age of (43.66 ± 3.60) years. All selected patients met the indications related to chemotherapy, and the following criteria were included: those who met the relevant diagnostic criteria; those who met the treatment indications; those who did not interrupt the treatment; those who did not have psychiatric disorders; and those who did not have serious psychological problems.

The study was reviewed by the medical ethics committee, and the following cases were excluded: those with combined schizophrenia; pregnant and lactating women; those with combined hematological and immune system diseases; those with combined systemic infectious diseases; and those with combined coagulation abnormalities.

### 2.2. Care Methods

Patients in the control group were given conventional nursing intervention mode, combined with the actual needs of patients, and given corresponding guidance to provide patients with chemotherapy treatment-related nursing cooperation. Patients in the observation group were given systematic dietary guidance as follows: communicate with patients, grasp their daily dietary habits, and help them analyze dietary contraindications during chemotherapy treatment. Communicate with the dietitian about the patient's situation, and jointly develop a good diet plan and program to meet the individual needs of the patient as much as possible, generally ensuring that protein accounts for about 60%, fat 25%, and a certain amount of carbohydrate intake. Chemotherapy treatment is more harmful to the patient's body and gastrointestinal adverse reactions are more common. The nursing staff instructs the patient to eat nutritious and non-stimulating food, such as chicken and milk, and try to eat in semiliquid form, which can ensure the adequacy of nutrient absorption and also reduce a variety of adverse reactions. Explaining the key points of post-discharge diet and informing precautions in conjunction with patients' physical condition strengthen patients' post-discharge compliance behavior and further improve patients' self-management ability.

In response to the patients' poor digestive symptoms, the causes of their occurrence are analyzed and different dietary care countermeasures are taken, including (1) loss of appetite, which is mostly caused by the effect of toxins brought about by tumor growth, thus the nursing staff should instruct the dietitian to pay attention to the color and aroma of food when caring for their diet in order to arouse patients' appetite. At the same time, patients can take a small amount of exercise before eating to promote gastric emptying and gastrointestinal peristalsis, and can also be given foods that strengthen the spleen and stomach to improve their appetite; (2) vomiting and nausea, which are mostly caused by the adverse effects of taking anticancer drugs, so patients should avoid eating as much as possible before receiving chemotherapy, and after receiving chemotherapy, they can take less and more meals to reduce the feeling of nausea brought by food digestion; (3) oral ulcers, which are caused by the reduction of granulocytes in the patient's body after receiving chemotherapy and the influence of bone marrow hematopoietic function, which makes the oral flora multiply and destroy the oral mucosa. For these patients, the intake of cold or hot stimulating food should be prohibited, and the mouth should be rinsed with hydrogen peroxide or mouthwash in time after eating to keep the mouth clean. Patients should be given vitamin B to improve ulcer symptoms; (4) constipation is mainly caused by reduced physical activity and slower gastrointestinal motility during treatment. To relieve constipation, patients can consume more vegetables and fruits and coarse fiber-rich cereals. At the same time, patients can drink more water to speed up the excretion rate of drugs in the body, and prohibit the consumption of spicy, yam, glutinous rice, and other intestinal food. Patients should be instructed to perform moderate exercise to promote the recovery of gastrointestinal motility; and (5) stomach discomfort, patients with clinical manifestations of indigestion, abdominal distension, etc. Such patients are mostly affected by gastrointestinal hypofunction, while caring, patients should be instructed to choose light and easily digestible food, adhere to a small number of meals, and prohibit the consumption of greasy fried food. Bifidobacterium can also be given to improve gastrointestinal function if necessary (Tables 1 and 2).

Environmental accounting implementation indicators in this paper are based on literature analysis, case study, and fuzzy comprehensive evaluation. This paper is different from previous studies on the implementation index of environmental accounting. In this paper, environmental accounting is divided into financial and nonfinancial information, and different scores are assigned to government subsidies and construction in progress depending on the number of projects, and environmental protection and greening costs include environmental protection costs and environmental maintenance costs.

### 2.3. Observation Items

Of the eight studies included in the literature [9–16], two [11] studies described the specific randomization method and process, while six [10–16] studies only described the randomization method used; four [11–15] studies reported the method of allocation scheme concealment, while the remaining four [10–16] studies did not specify; four [10–12] studies used double-blind and one [16] study used single-blind (blinded to the study population), while the rest did not describe it in detail; seven [10–15] studies reported the complete data results; one [16] study reported the complete data results; and one [16] study reported the complete data results. References [10–12] studies were double-blinded, one study was single-blinded (blinding of subjects), and the rest were not discussed in detail; seven [10–15] studies reported complete data results; one [16] study may have been selective; two [10–15] studies were designed rigorously to exclude other sources of bias The remaining studies may be at risk of other biases.

(1) Occurrence of gastrointestinal symptoms: statistical analysis of the occurrence of gastrointestinal symptoms in 36 patients before and after the nursing intervention; (2) Quality of life score: the quality of life of 36 patients before and after the nursing intervention was scored with a total score of 100, with higher scores indicating better quality of life [10]; (3) Nursing satisfaction: a questionnaire prepared by our hospital was used to compare the satisfaction of 36 patients before and after nursing care; (4) Satisfaction of nursing care: the satisfaction of 36 patients before and after nursing care was compared using our own questionnaire, in which satisfaction was divided into three levels, i.e., satisfied, basic satisfaction and dissatisfaction, and satisfaction of nursing care = (satisfied + basic satisfaction)/total number of cases × 100%.

## 3. Results

### 3.1. Effect of Dietary Intervention on Nausea and Vomiting

The incidence of nausea and vomiting was expressed as a dichotomous variable. Two [13, 14] studies used short-term (0 to 3 months) patient interventions, and one of them measured the effect on the control of nausea and vomiting in patients undergoing long-term (3 to 6 months) chemotherapy, and these studies were analyzed by subgroups according to the duration of the intervention. Dichotomous variables were used to express the incidence of nausea and vomiting, so RR values were calculated for the analysis. There was no heterogeneity among the studies (*P*=0.95, 12 = 0%), so a fixed-effects model was used for meta-analysis, and the results are shown in Table 3.

### 3.2. A Continuous Variable Was Used to Indicate the Frequency of Nausea and Vomiting

Three [10, 12, 15] studies indicated the effect of dietary care by the frequency of nausea and vomiting in patients during the intervention and were analyzed using standardized mean differences. There was heterogeneity among the studies (*P* < 0.0001, I2 = 93%), and sensitivity analysis concluded that the heterogeneity was probably due to the study of [15] and that the heterogeneity decreased from 93% to 0% after removing this study. A random-effects model meta-analysis was used, and the results are shown in Table 2. Three studies [10, 12, 15] expressed the effect of dietary care by the frequency of nausea and vomiting in patients during the intervention, and the analysis was performed using standardized mean differences. There was heterogeneity among the studies (*P* < 0.0001, I2 = 93%), and sensitivity analysis concluded that the heterogeneity was probably due to the study of [15], which was removed and the heterogeneity decreased from 93% to 0%. The results of the random-effects model meta-analysis are shown in Table 4.

### 3.3. Effect of Dietary Intervention on 4 Items of Quality of Life

The studies evaluated the impact of dietary care on chemotherapy patients' quality of life using the Quality of Life Assessment Scale, respectively, and subgroup analysis was performed by varying the duration of intervention in the above studies. In the short-term chemotherapy patients, there was excessive heterogeneity among the studies (*P* < 0.0001, 12 = 92%), and sensitivity analyses were performed, suggesting that the heterogeneity may have been due to the study by [16], and removing this study reduced the heterogeneity from 92% to 0%. The heterogeneity decreased from 92% to 0% after removing this study; there was no heterogeneity among studies in the long-term chemotherapy group (*P* = 0.16, 12 = 46%). The results of the random-effects model meta-analysis are shown in Table 5.

### 3.4. Impact on the Quality of Life of Chemotherapy Patients

The results of this systematic evaluation based on a meta-analysis of four [10, 11, 16] randomized controlled trials suggest that dietary care interventions have a positive effect on the quality of life improvement in chemotherapy patients. As shown in Figure 1, the long-term effect of dietary care on quality of life improvement is unclear compared to the short-term intervention effect, which may be related to the difficulty in maintaining the effect of nausea and vomiting control with prolonged chemotherapy cycles and the decline in the overall health status of patients, as recommended by the International Antiemetic Conference in Perugia [8], where benzodiazepines is currently used as an alternative therapy The synergistic effect of dietary interventions, especially in patients undergoing long-term chemotherapy, is not ideal, so the effect on improving the quality of survival of patients remains to be studied; the difference in the study results may also be related to the difference in sample size between the two groups.

## 4. Discussions

The results of this systematic evaluation based on 5 [10, 12–15] studies, using dichotomous and continuous variables, respectively, and a meta-analysis of short-term effects showed that dietary care reduced the occurrence of nausea and vomiting in chemotherapy patients in general, and the short-term effects were more pronounced. This may be related to the improved oral comfort of patients after the dietary intervention, improved knowledge of dietary care, and reduced damage to the gastrointestinal mucosa from chemotherapy. The effect of dietary interventions can be summarized as follows: firstly, to reduce nausea and vomiting by regulating the eating pattern; secondly, to improve the taste of food and thus the appetite of patients; thirdly, to protect the mucous membrane of the digestive tract by the active ingredients in food; regarding the specific mechanism of dietary care, scholars have already conducted studies on the pathway mechanism. The specific mechanism of dietary care has been studied from the perspective of pathways, and the specific mode of action of dietary care on the toxic reaction of the GI tract caused by chemotherapy has been elucidated from the biological point of view, which provides basic support for the clinical promotion of this measure and should be the direction of further development in the field of nursing in the future. A meta-analysis of 2 [13–15] randomized controlled trials showed that dietary care had a long-term effect on the relief of nausea and vomiting in patients undergoing long-term chemotherapy when dichotomous variables were used to indicate the control of nausea and vomiting. However, the long-term effect of dietary care on improving the adverse effects of nausea and vomiting in oncology chemotherapy patients when a continuous variable was used to indicate the effect of nausea and vomiting symptom control was unclear. This may be related, on the one hand, to the insufficient amount of literature included in this study; on the other hand, it may be related to the differences between the two studies in terms of ethnography and duration of intervention [19, 20].

In conclusion, dietary care has a positive effect on the improvement of nausea and vomiting symptoms and the quality of life of oncology chemotherapy patients, and the clinical management of the diet of oncology chemotherapy patients can be strengthened.

Some patients' glucose tolerance may also change abnormally during chemotherapy treatment, which may have a suppressive effect on patients' appetite. To address these reasons, in this study our nursing staff communicated with the dietitian to improve the patient's diet, paying attention to the color and flavor to stimulate the patient's appetite. Patients were also instructed to exercise before eating to accelerate gastric emptying and stimulate gastric acid secretion to increase their appetite. After the implementation of the care, the patient's symptoms of loss of appetite were significantly relieved. As for patients with stomach discomfort, which mostly occurs clinically, it is mainly caused by the reduction of gastrointestinal function due to the decrease of activity during treatment, and for such patients, the gastrointestinal function can be improved by appropriate exercise and improvement of the dietary structure, and bifidobacteria can be given if necessary, and aftercare, patients' discomfort such as indigestion and bloating basically disappeared, and gastrointestinal function was improved [11], and the incidence of various digestive symptoms This indicates that effective dietary care can improve patients' digestive system symptoms and reduce the occurrence of loss of appetite and gastric discomfort. At the same time, effective dietary care can also improve patients' satisfaction with care. From the results of this study, after receiving care, patients' satisfaction with care was significantly higher than before care, and patients' digestive reactions were reduced, which led to a substantial increase in patients' treatment comfort and tolerance of chemotherapy, thus improving satisfaction with care. From the results of this study, the incidence of gastrointestinal symptoms was significantly reduced, quality of life was significantly improved (59.92 ± 6.57) vs. (37.95 ± 7.50), and satisfaction with care was significantly higher (91.67% vs. 69.44%) in 36 patients after receiving care, and the results were basically consistent with those of [12], which proved that digestive symptoms in chemotherapy patients. This proves that dietary care plays an important role in the prevention and treatment of digestive symptoms in chemotherapy patients.

In conclusion, effective dietary care can effectively improve the digestive symptoms of chemotherapy cancer patients and reduce and prevent all kinds of digestive reactions, which is worth promoting in cancer clinical care.

## Figures and Tables

**Figure 1:** The dietary care intervention on the quality of life of chemotherapy patients.

**Table 1:** Comparison of the occurrence of gastrointestinal symptoms before and after care (*n* (%)).

Time	*n*	Loss of appetite	Nausea and vomiting	Mouth ulcer	Constipation	Stomach discomfort
Before nursing	36	33 (91.66)	6 (19.45)	12 (30.66)	7 (16.75)	22 (58.34)
After nursing	36	11 (30.66)	2 (2.79)	3 (12.11)	1 (2.78)	8 (19.45)
*x* ^2^		9.36	8.90	9.33	7.53	10.52
*P*		<0.05	<0.05	<0.05	<0.05	<0.05

**Table 2:** Comparison of patients' nursing satisfaction before and after care (*n* (%)).

Time	*n*	Satisfied	Basically satisfied	Dissatisfied	Nursing satisfaction
Before nursing	36	9 (25.00)	7 (44.45)	8 (30.66)	22 (69.45)
After nursing	36	23 (63.99)	10 (27.79)	3 (8.43)	34 (91.66)
*x* ^2^		10.37	8.20	9.37	8.53
*P*		<0.05	<0.05	<0.05	<0.05

**Table 3:** The effect of dietary care on nausea and vomiting (dichotomous variables).

Subgroup	RR (95% CI)	*P*
Short term (0∼3 months)	0.23 (0.10, 0.58)	0.003
Long term (3∼6 months)	0.25 (0.09, 0.72)	0.002

**Table 4:** The effect of dietary care on nausea and vomiting (continuous variables).

P	Subgroup	SMD (95% CI)
Short term (0∼3 months)	−0.99 (−1.28, − 0.67)	<0.001
Long term (3∼6 months)	−0.16 (−0.59, − 0.29)	0.52

**Table 5:** The effect of dietary care on quality of life.

Subgroup	SMD (95% CI)	*P*
Short-term (0∼3 months)	0.43 (0.15, 0.72)	0.005
Long-term (3∼6 months)	0.19 (−0.10, 0.45)	0.18

## Data Availability

The experimental data used to support the findings of this study are available from the corresponding author upon request.
